RETRACTED

# Effects of Fisetin on Allergic Contact Dermatitis via Regulating the Balance of Th17/Treg in Mice

**DOI:** 10.1155/2022/9222541

**Published:** 2022-04-09

**Authors:** Bocui Song, Xue Shen, Shuang Zhang, Rui Zhao, Yanhong Wang, Mengmeng Jiang, Min Liu, Qian Chen, Yuqi Li, Baolei Huang, Chenghao Jin, Chunyu Tong

**Affiliations:** ^1^Department of Pharmaceutical Engineering, College of Life Science & Technology, Heilongjiang Bayi Agricultural University, Daqing, 163319 Heilongjiang Province, China; ^2^Molecular Mechanism of Disease & Research and Development of Bioactive Substances, College of Life Science & Technology, Heilongjiang Bayi Agricultural University, Daqing, 163319 Heilongjiang Province, China; ^3^Animal Husbandry and Veterinary Station of Yongji Economic Development Zone, Jilin, 132200 Jilin Province, China; ^4^Department of Biological Engineering, College of Life Science & Technology, Heilongjiang Bayi Agricultural University, Daqing, 163319 Heilongjiang Province, China; ^5^Department of Biological Science, College of Life Science & Technology, Heilongjiang Bayi Agricultural University, Daqing, 163319 Heilongjiang Province, China

## Abstract

**Background:**

Allergic contact dermatitis (ACD) is a form of chronic cutaneous inflammatory disease of immunological origin that has adverse impacts on patient quality of life, underscoring the need for the development of safe and effective therapeutic agents to treat affected individuals. Fisetin is a Chinese herbal preparation that reportedly exhibits antitumor, antioxidant, antimicrobial, anticoagulatory, and antimalarial activity. In the current report, the immunomodulatory activity of fisetin was appraised by assessing its impact on balance between regulatory T (Treg) and Th17 cells in an ACD model.

**Methods:**

BALB/c mice (*n* = 60) were randomized into control, ACD model, CTX positive control (20 mg/kg), and fisetin treatment groups (three dose levels: 2, 4, or 8 mg/kg). ACD induction was achieved by sensitizing mice on the shaved ventral abdomen via the application of 5% DNFB (50 *μ*L) on days 1 and 2, followed by rechallenge in the right ear with 5% DNFB (20 *μ*L) on day 5. Beginning on day 1, immunized mice were intraperitoneally injected with the appropriate fisetin dose (in saline) once per day for 7 days. On day 7, ear swelling, transcription factor expression, Th17/Treg cell populations, and cytokine production were assessed in vivo.

**Results:**

Fisetin treatment significantly suppressed ear swelling and associated inflammatory cell infiltration, besides reducing the production of Th17 cytokines (IL-17, TNF-*α*, and IL-6) and the expression of the Th17 lineage transcription factor ROR*γ*t while simultaneously enhancing Treg-specific cytokine production (TGF-*β* and IL-10) and the expression of the Treg lineage transcription factor Foxp3, thereby restoring the Th17/Treg cell in ACD mice.

RETRACTED

**Conclusions:**

These data indicate that fisetin exhibits immunomodulatory activity and can alter the Th17/Treg cell balance, highlighting its potential value as a treatment drug for ACD.

## 1. Introduction

Allergic contact dermatitis (ACD) is a form of T cell-mediated inflammatory skin disease in which sensitized T cells react to particular antigens and release inflammatory cytokines, thereby promoting localized inflammatory cell infiltration, tissue degeneration, and necrosis [1–3]. Many reports have demonstrated a link between ACD incidence and an imbalance between the Th1 and Th2 CD4^+^ T cell subsets. Recent work further suggests that Th17 and regulatory T (Treg) cells can also modulate immune homeostasis [4–6].

ACD patients often experience symptoms such as pruritus, edema, erythema, and coalescing edematous papules [7, 8]. The World Health Organization estimates that 15% of the global population is affected by ACD. Topical treatments for ACD include nonsteroidal anti-inflammatory drugs, H1 receptor antagonists, and glucocorticosteroids. These drugs exhibit a wide range of side effects when used at high doses, however [9–11], underscoring the need for the development of novel ACD treatments of fewer side effects.

Herbal medicines have long been used to treat diseases. Given the wide distribution of herbal resources, their inexpensive nature, and the low levels of toxicity associated with herbal medicine-based therapies, they hold great promise as advantageous means of treating disease. Fisetin (3,7,3,4-tetrahydroxyflavone) is a flavonoid present within a range of fruits and vegetables including apples, onions, grapes, strawberries, and cucumbers at doses of 2-160 *μ*g/g [12, 13]. Fisetin has previously been shown to inhibit monoamine oxidase activity associated with the norepinephrine and serotonin systems, thus exerting antidepressant activity [14–16]. It has also been reported to stimulate cell signaling, thereby improving long-term memory [17]. Moreover, fisetin can alter signal transduction, suppress tumor cell proliferation, migration, and invasion, and promote apoptotic tumor cell death [18–22]. It also exhibits hepatoprotective and reparative efficacy in the context of hepatitis-related liver damage [23, 24], while also mitigating aflatoxin cytotoxicity [25]. The chemical structure of fisetin is as indicated.

We have previously found that fisetin can suppress the Th1/Th2 cell balance in vitro and in vivo in addition to suppressing IL-17 production, suggesting that this compound has the potential to modulate Th17 cell functionality. To more fully explore the immunopharmacological activity of fisetin, we herein assessed its ability to modulate the Th17/Treg balance and to thereby attenuate disease severity in a murine model of DNFB-induced ACD.

RETRACTED

## 2. Materials and Methods

### 2.1. Chemicals and Reagents

Fisetin (>98% pure, catalog number: 528483, Figure 1) was obtained from Sigma-Aldrich and diluted in culture media containing 0.1% DMSO, sterile filtered, and stored at 4°C prior to utilization. An equivalent DMSO concentration was used for all control animals. Cyclophosphamide (CTX) and 2,4-dinitrofluorobenzene (DNFB) were procured from Sigma (MO, USA). RPMI-1640 was from HyClone (Logan, UT). Moreover, BioLegend (CA, USA) supplied IL-6, IL-17, TGF-*β*, TNF-*α*, and IL-10 ELISA kits. PE-anti-IL-17A, FITC-anti-CD4, APC-anti-CD25, and PE-anti-Foxp3 were from BD Pharmingen.

### 2.2. Animals

BALB/c mice (16-18 g, 6-8 weeks old, 50% male, 50% female) were acquired from the Jilin University Experimental Animal Center and housed in microisolator cages with free water and food accessibility. The Animal Welfare and Research Ethics Committee at Heilongjiang Bayi Agriculture University approved all animal studies.

### 2.3. ACD Model Establishment

To induce ACD, the ventral abdomen of mice was shaved and sensitized with 5% DNFB (50 *μ*L; acetone : olive oil = 4 : 1) on days first and second. After five days, mice were then challenged through painting both the outer and inner surfaces of the right ear with 10 *μ*L of 5% DNFB (acetone : olive = 4 : 1), while the left ear was painted with an equivalent volume of a control acetone and olive oil (4 : 1) mixture. Ear swelling at 48 h after the second challenge was then assessed by weighing ear patches from both ears prepared with an 8 mm punch and comparing these relative weights.

### 2.4. Drug Treatment

BALB/c mice (*n* = 60) were randomized into six groups (10/group) including a control group, an ACD model group, a positive control CTX (20 mg/kg) group, and three fisetin groups (2, 4, and 8 mg/kg). Treatments were intraperitoneally administered to mice once per day for 7 days, with control animals being administered an equivalent volume of 0.1% DMSO.

### 2.5. Ear Swelling Analyses

At 24 h post-DNFB stimulation, both ears were punched and the removed tissue was weighed as a means of quantifying ear swelling in these animals as a readout for the magnitude of ACD reactions as follows: 24 h after the mice were finally stimulated with DNFB for allergy, the left and right ears of the mice were punched and weighed to calculate the ear swelling of the mice, which reflects the reaction intensity of ACD. Formula: edema rate (mg) = *W*_right_ ear − *W*_left_ ear, where edema rate corresponds to ear swelling, *W*_right_ ear corresponds to right ear weight (mg), and *W*_left_ ear corresponds to left ear weight (mg).

RETRACTED

### 2.6. Histological Observations

At 24 h post-DNFB stimulation, the left and right auricles were collected using clean scissors from mice in each group and fixed for 24 h in 10% formalin. These tissues were then dehydrated, inserted in paraffin, and cut into segments. Following deparaffinization, hematoxylin-eosin staining was performed and tissues were imaged via microscopy to identify appropriate representative regions for analysis.

### 2.7. Flow Cytometry

On day 7 of the study period, 1 × 10^6^ splenocytes were rinsed with PBS, after which red blood cells were lysed employing ACK lysis buffer and the left lymphocytes were suspended in RPMI-1640 including 10% FBS. Th17 and Treg cells were analyzed through incubating these cells for 4 h with ConA and then staining them with PE-anti-IL-17A, FITC-anti-CD4, APC-anti-CD25, and PE-anti-Foxp3 followed by subsequent flow cytometry-based quantification.

### 2.8. Analysis of Foxp3 and ROR*γ*t mRNA Level Expression

TRIzol was employed for the extraction of total RNA from splenocytes, following which a RevertAid first-strand cDNA synthesis kit and random primers were used to synthesize cDNA. Then, SYBR® Premix Ex Taq™ II was used to amplify the Foxp3, ROR*γ*t, and *β*-actin in a 25 *μ*L reaction volume, with *β*-actin serving as a normalization control. Primer sequences employed in this research are compiled in Table 1.

### 2.9. ELISAs

Capture antibodies were incubated in 96-well plates overnight at 4°C, after which plates were washed and 100 *μ*L of appropriate blood samples was added to appropriate wells, succeeded by a 2 h incubation at 37°C. Plates were then rinsed 4 times, succeeded by the addition of 100 *μ*L of secondary antibody (1 : 200) at 37°C for 1 h. Plates were then rinsed again and incubated by implementing 100 *μ*L of horseradish peroxidase (HRP; 1 : 1000) per well at 37°C for 30 min. Plates were subsequently rinsed 5 times using wash buffer, and 100 *μ*L of TMB substrate was then added per well. Following a 15 min incubation at 25°C while protected from light, reactions were terminated via the addition of 2 M H_2_SO_4_. Plates were then allowed to stand for 5 min, after which a microplate reader was used to assess OD values at 450 nm. A standard curve was then used to measure IL-17, IL-10, IL-6, TNF-*α*, and TGF-*β* content in each sample.

### 2.10. Statistical Analyses

Data are means ± standard deviations (SD) and were compared via Student's *t*-test employing SPSS 13.0. *P* < 0.05 was the significance threshold (*n* = 3).

RETRACTED

## 3. Results

### 3.1. Fisetin Suppresses Ear Swelling in a Murine ACD Model

Relative to the control group, ear swelling in ACD model mice was substantially enhanced (*P* < 0.01; Figure 2(a)), while following the intraperitoneal injection of fisetin, analyses revealed that a low fisetin dose significantly suppressed ear swelling in these animals (*P* < 0.05), with medium and high fisetin doses having an even more pronounced inhibitory effect of such swelling in a dose-dependent manner (*P* < 0.01). Low-dose fisetin treatment was more efficacious than treatment with the clinical immunosuppressive drug CTX.

### 3.2. Fisetin Normalizes Histopathological Findings in ACD Model Mice

To more fully evaluate the impact of fisetin treatment, ear tissue sections from treated mice were subjected to H&E staining. Relative to control animals, those in the ACD model group demonstrated increased inflammatory cell infiltration and swelling following DNFB challenge, consistent with successful ACD model establishment (Figure 2(b)). However, fisetin treatment significantly reduced such inflammatory infiltration relative to the ACD and CTX groups, further confirming the ability of fisetin to suppress ACD-related ear swelling.

### 3.3. Fisetin Modulates the Th17/Treg Balance in ACD Model Mice

The impact on fisetin treatment of Th17 and Treg cell populations in ACD model mice was next assessed (Table 2). Relative to control animals, ACD model mice exhibited significant increases in Th17 cells and substantial reductions in Treg cells (*P* < 0.01), whereas fisetin and CTX treatment reversed these alterations (*P* < 0.05 or *P* < 0.01). The obtained outcomes define that fisetin is capable of regulating the Th17/Treg cell balance.

### 3.4. Fisetin Modulates ROR*γ*t and Foxp3 mRNA Expression in ACD Model Mice

Next, RT-PCR was employed to appraise relative ROR*γ*t and Foxp3 expression in splenocytes. Relative to control animals, ACD model mice exhibited increased expression of the Th17-specific transcription factor ROR*γ*t and decreased expression of the Treg-specific transcription factor Foxp3 at the mRNA level (*P* < 0.01, Figure 3). Following fisetin or CTX treatment, ROR*γ*t mRNA levels were substantially diminished, while Foxp3 levels were enhanced with respect to the ACD model group (*P* < 0.01).

### 3.5. Fisetin Modulates Cytokine Production in ACD Model Mice

Next, serum IL-17, IL-10, IL-6, TNF-*α*, and TGF-*β* levels in these ACD model mice were assessed via ELISA (Figure 4). Relative to controls, ACD model mice exhibited enhancements in TNF-*α*, IL-6, and IL-17 levels (*P* < 0.01), while TGF-*β* and IL-10 levels were significantly reduced in these ACD model mice (*P* < 0.05 or *P* < 0.01). Conversely, fisetin and CTX treatments reduced TNF-*α*, IL-6, and IL-17 levels (*P* < 0.05 or *P* < 0.01) while increasing TGF-*β* and IL-10 levels (*P* < 0.05 or *P* < 0.01). The obtained outcomes illuminate that fisetin is able to suppress inflammatory cytokine production while enhancing the secretion of anti-inflammatory cytokines.

RETRACTED

## 4. Discussion

Allergic contact dermatitis is a relatively common form of allergic skin disease that can be triggered by sensitizing allergens which can be challenging to avoid in daily life. ACD treatment at present primarily relies on the use of H1 receptor antagonists and glucocorticoids, but these exhibit relatively limited efficacy and high rates of side effects [26–28], highlighting a need for the design of novel, safe treatments for this condition. Fisetin is a flavonoid compound present within a variety of plants, fruits, and vegetables [29, 30]. We have previously shown fisetin to suppress Th1/Th2 cell activities, and we herein sought to expand these analyses by assessing its ability to modulate Th17/Treg immunological homeostasis in a murine model of ACD [31, 32].

Repeated DNFB application successfully induced a model of ACD in our experimental mice characterized by pronounced ear swelling by 48 h post-DNFB application. Fisetin treatment was sufficient to alleviate such swelling, and these findings were further confirmed through histopathological analyses revealing that fisetin was able to reduce DNFB-induced epidermal inflammation and inflammatory cell infiltration.

CD4^+^ Th17 and Treg cells exhibit opposite performances in the regulation of autoimmune inflammation and the maintenance of immune homeostasis [33, 34]. Prior work suggests that excess Th17 cell activation and impaired Treg activity are correlated with the expansion of a range of autoimmune disorders. As such, modulating this Th17/Treg balance may effectively treat ACD [35, 36]. We thus explored the capability of fisetin for modulating the Th17/Treg balance in our ACD model mice. While ACD model animals exhibited increases in Th17 cells and decreased Treg cell levels relative to controls, fisetin and CTX treatment decreased Th17 cell frequencies and enhanced Treg cell frequencies. These data suggest that Th17/Treg cell imbalance is a hallmark of ACD that is amenable to fisetin-mediated immunomodulatory regulation.

ROR*γ*t and Foxp3 are lineage-specific regulatory transcription factors that control the function and differentiation of Treg and Th17 cells, respectively [37, 38]. To assess the ability of fisetin to alter the expression of these transcription factors, we examined Foxp3 and ROR*γ*t expression in ACD model mice, revealing that such treatment reduced decreased ROR*γ*t expression and enhanced Foxp3 expression. As such, these data support the existence of Th17/Treg imbalance in ACD model mice that was remediated by fisetin treatment.

RETRACTED

Cytokines function as key regulators of the differentiation of Th17 and Treg subsets, with IL-6 and TGF-*β* modulating the expression of lineage-specific transcription factors within CD4^+^ cells in the context of such fate determination [39, 40]. Low TGF-*β* concentrations in the presence of IL-6 are able to drive the differentiation of Th17 cells and their consequent secretion of IL-17A and TNF-*α*, which in turn promote local inflammation, whereas high TGF-*β* concentrations are capable of promoting the differentiation of Tregs [41, 42]. IL-10 is an anti-inflammatory cytokine that hinders inflammatory cell activation and proinflammatory cytokine secretion [43, 44]. Here, we found that fisetin treatment was associated with marked reductions in IL-17A, IL-6, and TNF-*α* treatment relative to the levels of these cytokines in ACD model mice, whereas the Treg-related cytokines IL-10 and TGF-*β* were present at high levels in fisetin-treated mice. This suggests that fisetin can suppress ACD-related disease pathology by enhancing anti-inflammatory IL-10 and TGF-*β* production while downregulating levels of inflammatory mediators including IL-17A, IL-6, and TNF-*α*.

Briefly, we herein employed a DNFB-induced murine ACD model system to demonstrate that fisetin treatment was sufficient to suppress ear swelling following DNFB treatment owing to its ability to inhibit the recruitment of inflammatory cells to the inflamed ear tissue section. Fisetin was also able to restore the Th17/Treg balance in these mice by inhibiting the secretion of IL-17, IL-6, and TNF-*α* and the expression of ROR*γ*t at the mRNA level while enhancing TGF-*β* and IL-10 secretion and promoting the mRNA-level upregulation of Foxp3. Fisetin may thus represent a viable candidate drug for ACD treatment owing to its ability to modulate the Th17/Treg balance.

## Figures and Tables

**Figure 1:** The chemical structure of fisetin.

**Figure 2:** Fisetin treatment reduces allergy-related ear thickness. (a) Ear thickness measurements and (b) histopathological analyses in a murine ACD model. Increases in the weight of 8 mm ear punch tissue sections were used to analyze ACD reaction severity by comparing the right and left ears at 48 h following a second challenge. Histological alterations in the right ears of these mice were assessed at 48 h after DNFB treatment (200x). Data are means ± SD (*n* = 3). ^##^*P* < 0.01 vs. control group. ^∗^*P* < 0.05 and ^∗∗^*P* < 0.01 vs. ACD group.

RETRACTED

**Figure 3:** Fisetin alters ROR*γ*t and Foxp3 mRNA expression *in vivo*. (a) Representative electrophoretic analysis results for RT-PCR products. (b) The ratio of relative ROR*γ*t or Foxp3 expression was quantified through a densitometric pathway, with *β*-actin being employed for normalization. Data are means ± SD (*n* = 3). ^##^*P* < 0.01 vs. control group. ^∗^*P* < 0.05 and ^∗∗^*P* < 0.01 vs. ACD group.

**Figure 4:** Fisetin alters cytokine production. ELISAs were used to measure serum levels of (a) IL-17, (b) IL-6, (c) TNF-*α*, (d) TGF-*β*, and (e) IL-10 at 48 h following the second challenge. Data are means ± SD (*n* = 3). ^##^*P* < 0.01 vs. control group. ^∗^*P* < 0.05 and ^∗∗^*P* < 0.01 vs. ACD group.

**Table 1:** Primers employed for PCR.

Primer	Sequence
Foxp3	5′-TTTCACCTATGCCACCCTTATC-3′ 5′-GTAGGCGAACATGCGAGTAA-3′
ROR*γ*t	5′-ACCTCCACTGCCAGCTGTGTGCTGTC-3′ 5′-TCATTTCTGCACTTCTGCATGTAGACTGTCCC-3′
*β*-Actin	5′-CCCATCTATGAGGGTTACGC-3′ 5′-TTTAATGTCACGCACGATTTC-3′

**Table 2:** The impact of FIS on Th17/Treg of ACD mice.

Group	Treg (%)	Th17 (%)	Th17/Treg (%)
Control	9.672 ± 0.781	0.581 ± 0.014	0.064 ± 0.013
ACD	7.013 ± 0.269^##^	2.805 ± 0.293^##^	0.412 ± 0.016^##^
CTX	8.201 ± 0.105	1.394 ± 0.093^∗∗^	0.175 ± 0.038^∗∗^
Fisetin 2 mg/kg	7.828 ± 0.484^∗^	2.739 ± 0.102	0.354 ± 0.023
Fisetin 4 mg/kg	8.565 ± 0.677^∗∗^	1.799 ± 0.203^∗∗^	0.219 ± 0.039^∗∗^
Fisetin 8 mg/kg	9.283 ± 0.371^∗∗^	1.272 ± 0.322^∗∗^	0.143 ± 0.034^∗∗^

Notes: ^##^*P* < 0.01 vs. control group. ^∗^*P* < 0.05 and ^∗∗^*P* <0.01 vs. ACD group.

## Data Availability

The data used to support the findings of this study are available from the corresponding author upon request.
